# Advances in S gene targeted genome-editing and its applicability to disease resistance breeding in selected *Solanaceae* crop plants

**DOI:** 10.1080/21655979.2022.2099599

**Published:** 2022-07-26

**Authors:** Geleta Dugassa Barka, Jundae Lee

**Affiliations:** a Department of Horticulture, Institute of Agricultural Science & Technology, Jeonbuk National University, Jeonju, South Korea; b Department of Applied Biology, School of Applied Natural Science, Adama Science and Technology University, Adama, Ethiopia

**Keywords:** Susceptibility, *solanaceae*, mutagenesis, effector, pathogenicity

## Abstract

Genome-editing tools for the development of traits to tolerate abiotic and biotic adversaries are the recently devised breeding techniques revolutionizing molecular breeding by addressing the issues of rapidness and precision. To that end, disease resistance development by disrupting disease susceptibility genes (S genes) to intervene in the biological mechanism of pathogenicity has significantly improved the techniques of molecular breeding. Despite the achievements in genome-editing aimed at the intervention of the function of susceptibility determinants or gene regulatory elements, off-target effects associated with yield-related traits are still the main setbacks. The challenges are attributed to the complexity of the inheritance of traits controlled by pleiotropic genes. Therefore, a more rigorous genome-editing tool with ultra-precision and efficiency for the development of broad-spectrum and durable disease resistance applied to staple crop plants is of critical importance in molecular breeding programs. The main objective of this article is to review the most impressive progresses achieved in resistance breeding against the main diseases of three *Solanaceae* crops (potato, *Solanum tuberosum*; tomato, *Solanum lycopersicum* and pepper, *Capsicum annuum*) using genome-editing by disrupting the sequences of S genes, their promoters, or pathogen genes. In this paper, we discussed the complexity and applicability of genome-editing tools, summarized the main disease of *Solanaceae* crops, and compiled the recent reports on disease resistance developed by S-gene silencing and their off-target effects. Moreover, GO count and gene annotation were made for pooled S-genes from biological databases. Achievements and prospects of S-gene-based next-generation breeding technologies are also discussed.

## Highlights

- Most S genes are membrane –anchored and are involved in infection and pre-penetration process
- S gene-editing is less likely to cause an off-target effect
- Gene-editing has been considered a more acceptable engineering tool
- Editing S genes either from the pathogen or host ends has opened new possibilities

## Introduction

The family *Solanaceae*, one of the highly diversified plant families, comprises 3000–4000 species, of which only a few are improved and exploited as crop plants in a wide range of agro-ecologies [1,2]. It includes the most cultivated and economically significant crop species subfamily Solanoidae, which comprises four genera (Solanum, Capsicum, Physalis, and Lycium) [3]. The production and consumption of vegetables, despite their less production by volume, is becoming an important part of agricultural produce due mainly to intensive agricultural practices. Essentially, they (along with other vegetables) make an important part of the human diet as food and nutrition securities remain pressing concerns worldwide. Five times serving per day of fruits and vegetables has been reported to significantly decrease premature death and mortality caused by chronic diseases [4]. Compounded with population growth, continuously increased demand for vegetables and incomes of urban and suburban inhabitants have led to the diversification of diet [5]. Among the vegetable crops, potato, tomato, and pepper are accounted for vegetables whose production and consumption are steadily increasing with a gross production value of above USD 184,209 in 2016 (http://www.fao.org/faostat/en/#data/QV).

Unlike cereal crops, vegetables are generally considered the sources of many pathogenic microorganisms as raw vegetable consumption is preferable, mainly due to their rich nutritional composition when consumed uncooked. The nutritious and succulent nature of most vegetables also makes an ideal environment for the proliferation and cross-pathogenicity of microbes even during post-harvest storage. It was estimated that significant post-harvest loss in vegetables, as high as 36%, is caused by soft rot bacteria whose sources could be from the field, water used for cleaning, processing equipment and during storage [6]. Besides significant loss to diseases, microbes are also the causes of deteriorations of the quality of vegetables which impacts the price and consumer demand. Consumed around the world and steadily penetrating the fast-food industries’ supply chain, post-harvest management of potato, tomato, and pepper is decisively important to tap the utmost profit from their sustainable production. Post-harvest spoilage of vegetables is often caused by bacteria, fungi, and viruses though few of the diverse types of microbial species show host preference. Among the microbial species accounted for targeting a wide range of vegetables include *Botrytis cinerea Colletotrichum, Alternaria, Cladosporium, Phytophthora*, and *Rhizopus* spp. inflicting compromised quality and devastating post-harvest losses of vegetables with linked implications to cause food-borne illness to humans in some cases [7].

Feeding the ever-increasing population is putting an unprecedented burden on plant breeders to improve food production and minimize post-harvest loss. It requires more precise breeding techniques, which substantially minimize the time required for higher production volume. The most recently devised breeding technique revolutionizing molecular breeding to address the issue of rapidness and precision is genome-editing for the development of traits to tolerate abiotic and biotic stresses. Among the others, disease resistance breeding by disrupting disease susceptibility genes to intervene in the biological mechanism of pathogenicity has been the breakthrough vis-à-vis random mutagenesis and the conventional genetic transformation for resistance development [8,9]. Classical breeding (where disease resistance genes are introduced to elite plant materials), marker-assisted breeding, and genetic transformation were breeding tools behind the advancements of resistance breeding in the last two or so decades. Despite the achievements so far, the less precise, random, and bulk genetic recombination has been considered cumbersome in terms of precision and rapidness and hence an alternative breeding strategy, genome-editing-based breeding, targeting susceptibility genes, has been at the forefront in resistance breeding. A plant gene that supports microbial infection and facilitates its compatibility with the pathogen is referred to as susceptibility (S) gene.

The concept of resistance development by mutating susceptibility genes is an emerging resistance breeding approach by which overlapping roles of some genes, such as resistance and susceptibility factors, are exploited in some plants [10]. As more insights into resistance mechanisms are enabling the rapid development of disease resistance by susceptibility-based genome-editing, this approach has been considered as the most rampant and efficient tool for resistance breeding. The development of disease resistance by genome-editing of susceptibility conditioning genes (by disrupting the gene or promoter sequences) has been increasingly deployed in several crop plants as editing precision is achieved by the advent of CRISPR (clustered regularly interspaced palindromic repeats), ODM (Oligonucleotide-directed mutagenesis), TALE (transcription activator-like effector), and ZF (zinc-finger) nucleases-based site-directed mutagenesis. The applicability of these techniques has been proven to be promising in many staple crops and vegetables for the development of disease resistance against the most pressing disease-causing pathogens including viruses [11].

Despite the great leaps in the successful genome-editing aimed at the intervention of the function of susceptibility determinants or gene regulatory elements, off-target effects that adversely impact yield-related traits are still the main setbacks. The challenges are attributed to the complexity of the inheritance of traits controlled by pleiotropic genes. As the application and the versatility of multiple genome-editing techniques are being devised for disease resistance development in different crops, it would be certain that molecular breeding in vegetables (as it would be for cereal crops, too) will see a more rigorous, precise, and efficient in terms of time required and resource expenditure compared to traditional breeding. As different variants of gene editing are being refined and novel ones are being developed, an up-to-date compiled review could provide valuable insights for further advancements in S gene-based genome-editing applied to disease resistance breeding. Despite its increasing acceptances compared to classical genetic engineering, S gene-editing technologies for the development of disease-resistant *Solanaceae* crops are in their infancy, and the availability of such scientific reports is limited. Recent reports in potato on the development of late blight resistance using RNAi- and CRISPR/Cas9-based S-gene editing have shown promising results that could be applied to other crops as well [12,13]. The advancements in the approaches and precisions for manipulating S-genes are therefore worth compiling as they are less understood and limited in availability for a better understanding of the mechanism of resistance development and its applications in crop plants. To that end, the main objective of this review is to discuss the most recent and impressive progress in resistance breeding against the main pathogens in three *Solanaceae* crops (potato, tomato, and pepper) using genome-editing by disrupting the sequences of susceptibility genes, or promoters or genes of the pathogen. We also discuss some of the limitations from the latest reports on the achievements and future prospects of next-generation breeding based on the different approaches of S-gene editing and bioinformatics tools.

## Genome-editing: mechanisms and variant tools

The isolation and characterization of the first restriction nuclease from *Haemophilus influenza* [14] for the purpose of specific cutting of DNA nucleotide has paved the way for the development of fundamentally different tools of genetic engineering with better precision and speed of genetic manipulation. Genome-editing is a technique by which DNA mutations in the form of insertion and/or deletion (indels) or base substitutions are introduced to create an organism with a new or modified product. Central to the current advancements in genome-editing applied to plant genetic improvement was the knowledge acquired from the investigations into bacterial and viral biochemistry and molecular genetics for the manipulation of DNA, vector systems, and DNA delivery tools into cells. One of the milestones was the introduction of targeted local mutagenesis and incorporation of homologous donor sequences by intentional introduction of double-strand breaks (DSBs) using a rare-cutting meganuclease I-SecI [15]. Since then, the discovery of novel nucleases and the modification of the existing nucleases to catalyze DSBs at a precise site in the genome have further enhanced the modification of DNA at the target site. Cleavage and rejoining of DNA on specified sites is possible by the use of engineered nucleases as tools to modify the hereditary unit of a cell. In all the currently utilized genome-editing tools, the challenges in editing complex genomes such as polyploid genomes are designing multi-domain chimeric nucleases with the capability of selectively binding to specific DNA sequences and catalyzing the DNA cleavage at that site [16]. Such chimeric nucleases are also designed to be produced inside the target cell following the delivery by plasmid vectors with nuclear localization signal or direct introduction to the genomic DNA for their sustained integration into the host cellular gene expression system. In a recent report [17], variants of synthetic chimeric nucleases with improved precision and specificity that function in bacteria, yeast, and human cell lines have been developed. The delivery of a nuclease-based genome-editing system could be a direct physical method or vector-based delivery of mRNA or DNA, and exhaustive reviews for different host systems are available [18,19]. Among the couples of genome editing approaches, mechanisms, and tools, the most frequently used ones are discussed below.

### Zinc-finger nuclease-based genome-editing

Zinc-finger nucleases (ZFNs) are the first synthetic restriction enzymes with DNA-binding domains that specifically bind three base pairs at the target site, revolutionizing DNA manipulation in eukaryotes [20]. The structure of ZFN is composed of a site-specific Cys2-His2 zinc finger DNA binding domain fused with a non-sequence-specific DNA cleavage FokI (from *Flavobacterium okeanokoites*) domain [21]. Each ZFN monomer constitutes 30 amino acids arranged in two anti-parallel β-sheets opposing the α-helix [22]. The ZFN monomers bind to a specific three base pair sequence flanking 5-6-base pairs spacer on the target sequence via the α-helix unit which subsequently allows the cleavage in the major groove DNA by the FokI dimer within that spacer sequence [23,24]. The functional specificity lies in the 3–6 Cys2-His2 array of zinc finger domain which could be customized to target a specific sequence of interest on the target sequence [25]. In such approach, custom-DNA binding ZFNs could be engineered using the modular structure of zinc finger protein frameworks for the recognition and cleavage of a larger base pair DNA sequence. The linkage of the pre-selected ZFN module could potentially target the 64 nucleotide triplets in tandem to recognize the DNA sequence containing a series of specific triplet nucleotides [23]. Gene manipulation by ZFN involves the introduction of targeted DSB that stimulates cellular DNA repair mechanisms with a concomitant mutation. The endogenous DSB repairing machinery fixes the breaks either by non-homologous end joining (NHEJ) or homologous recombination repair (HR) [24]. When dsDNA is linked to the ZFN system, the repair would be homologous recombination (HR) while the random introduction of mutation (indel/substitution) by non-homologous end joining (NHEJ) would ultimately lead to the introduction of frameshift mutation to the target gene sequence. It was also reported that zinc finger nickase system errors and off-target effects were minimum as the homology-directed repair (HDR) was favored over NHEJ, further increasing the precision of ZFNs mediated genome-editing [26]. The advantages of ZFNs based genome-editing over the other tools with respect to efficiency, specificity, and off-target effects in addition to the current improvements have further entrenched its wider application in crop improvement [16]. Moreover, the smaller size of ZFN expression elements relative to the expression elements of TALENs and CRISPR/cas systems makes ZFN tools more suitable for viral vector-based delivery of the expression elements [27]. However, owing to the complexity of ZFNs-based engineering and the difficulties in multiplexing, the application of ZFN-based genome-editing has little impact on crop improvement for disease resistance [28]. A more applicable ZFN-based disease resistance development was attainable in targeting pathogenic viruses. The use of artificially designed zinc finger proteins has successfully demonstrated resistance against beet severe curly top virus [29], begomovirus [30] and tomato yellow leaf curl [31] by blocking DNA binding sites of viral replication proteins.

### TALEN-based genome-editing

The search for a more efficient and precise tool for DNA manipulation has lead to the identification and modification of TALE proteins from *Xanthomonas* bacteria [32] that bind to a specific sequence of the promoter for the activation of the downstream gene. Further characterization of TALEs revealed the role of tandem repeats for the specificity of the protein domain based on which the development of chimeric genome-editing tool known as transcription factor-like effector nucleases (TALENs) was developed [33]. TALENs are comprised of two domains: a nonspecific DNA cleaving domain that cleaves DNA in a nonspecific manner that is fused to a DNA binding domain which could be engineered so that virtually any kind of sequence binding is possible [34]. The engineering of TALENs for various genome-editing objectives has come from the characterization of TALE proteins involved in gene expression. As the DNA binding domain of TALEs is of critical importance in the eventual development of TALENs by genetic engineering, the decoding of the target DNA recognition sequence that signals the binding of DNA binding domain [35] revealed the central repeat domain (CRD) with a tandem repeat of 34 amino acid residues for DNA binding and host specificity [16]. A super variable repeat residue at the 12 and 13 amino acids of the tandem repeat forms repeat variable diresidue (RVD) for the recognition of specific nucleotides and a potential degeneracy to bind different nucleotides with different efficiency. The RVDs provide a structural feature to design and assemble variants of TALEN for a predictable DNA-binding role to induce any mutation of interest once delivered into the target cell. The half-repeat of the 20 amino acids, unlike the other 16 TALE repeats with 34 amino acid residues each, bind to the 3’-end of the target DNA and the conserved 5’-end thymidine binding TALE proteins determine the efficacy of TALE-transcription factors, TALE-recombinases and TALE-nucleases [34,36]. As reviewed by Joung and Sander [34], nucleotide specific binding of the TALE repeats domain precedes the ultimate nonspecific cleavage of target DNA catalyzed by FokI nuclease dimer domains of the C- and N-terminals at a spacer sequence flanking the specific target nucleotides. Since the identification of FokI, the nonspecific cleavage function of this domain has been fused to the specific nucleotide binding TALE repeat domains for the construction of chimeric nucleases to manipulate DNA for such purposes including genome-editing using variant editing tools [37]. Theoretically, DSB of DNA could be triggered at any site on the target DNA as far as it harbors the 5’-thymidine before the intended cleavage site. The constraint due to the 5’-thymidine requirement flanking the target sequence has been overcome by developing mutant TALENs, where N-terminal domain has been engineered to recognize other nucleotides at the 5’-end of the target sequence [36]. In their latest application as genome-editing tools, TALENs are used to either introduce random mutations, ssDNA- or dsDNA-guided alterations into the target genome following the creation of DSB at the target locus. The repair of DSB routes take different pathways depending on the nature of the introduced mutations; NHEJ to introduce random mutations (indel/substitution), homology-directed repair (HDR) for single-stranded template DNA-based repair and HR to introduce dsDNA into the target genome [25]. Error-prone NHEJ is designed for gene knockout by disrupting the coding sequence of that target gene due to the introduction of random indels or frameshift mutations while HDR and HR repairs are programmable and their effects are predictable. A more precise error-prone repair mechanism alternative to HR, microhomology-mediated end joining (MHEJ), has been believed to enhance the efficiency of genome editing in plants [38]. The mechanism of TALEN-based genome-editing is basically via the disruption of the effector-binding element of the S gene promoter which eventually impairs the compatible molecular interactions between the effector and the target S gene. It has been demonstrated that editing promoter regions of different variants of sugar transporter genes (SWEET genes), S gene, using TALENs, has resulted in the development of bacterial blight-resistant rice plants [39–41]. Despite the decreased efficiency in introducing sequence-specific mutations to the target plant S genes when compared to the one achieved using CRISPR/Cas9, resistances against begomoviruses have resulted in promising results in *N. benthamiana* [42].

### Oligonucleotide-directed mutagenesis

Oligonucleotide-directed mutagenesis (ODM) is another tool of genome-editing in which 20 to 100 base pair long nucleotide sequences are identical to the target sequence (except in a single nucleotide), where the intended point mutation is required. Oligonucleotide directed host DNA repair system introduces a mutation that disrupts the function of the target gene. The latest version of ODM is known as chimeraplasty, a technique in which an RNA/DNA chimeric nucleotide is used to introduce site-directed genomic alterations in plants [43]. A chimeraplast construct is composed of DNA and 2’-O-methyl-modified RNA designed to form a duplex region by complementary base pairing. The introduction of the synthetic oligonucleotide or template DNA (chimeraplast) to the target cell results in binding with the target sequence of homology except at a single mismatch, triggering the copying of that mutation into the target sequence through the base repairing process [16]. Integration of the synthetic chimeraplast into the target genome is prevented by the 3’- and 5’-end modifications and immediate degradation by host nuclease enzymes following the dissociation of the oligonucleotide from the target sequence [44]. The chimeric oligonucleotide consists of DNA, RNA, and end-protective chemistries that prevent recombination but still act as a mutagen and DNA template [45]. The process introduces the desired targeted single nucleotide mutation into the target genome resulting in the expression of a novel trait or function following the subsequent regenerations by plant tissue culture techniques and classical breeding [46]. Polyethylene glycol (PEG) and biolistics are the commonly used oligonucleotide delivery methods though the conversion rates depend upon different factors, such as crop type, cell biology system, oligonucleotide type, and concentration, the strand being targeted (sense or antisense) and the targeted mutation being made [45]. The application of ODM in precise genome-editing in models and different crop plants [45] for metabolic engineering, mode of action, as well as safety regulatory issues were reviewed by Songstad et al. [44]. Among the advancements in the ODM-mediated genome-editing in plants were the development of herbicide tolerance in canola [47], maize [48] and tobacco [49].

### CRISPR/Cas-based genome-editing

Since the discovery as an adaptive immunity in *Escherichia coli* [50] and later in many prokaryotes, CRISPR/Cas-based genome-editing has been increasingly adopted to manipulate the genome of many crop plants for different breeding objectives [16,42]. Despite the still unknown functions of most CRISPR-associated protein (Cas) types, they are broadly classified into two classes (class I and II), both classes comprise three types each (Class I includes types I, III, and IV; class II includes types II, V, and VI) [51]. Class I systems are the most abundant as they comprise about 90% of the CRISPR-Cas systems and are believed to have evolved earlier [52]. The multisubunit protein complexes with multiple Cas proteins of the class I systems are so crucial to cleave dsDNA, ssDNA and RNA for manipulation of cellular activities [53]. Class II comprises the type II Cas that in turn includes the most popular Cas9 nuclease identified from the bacterium *Streptococcus pyogenes* [16], Cas12a of type V [54] and Cas13a of type VI [55]. The type II CRISPR/Cas9 system is an RNA-guided exogenous sequence recognition and cleavage machinery that provides acquired immunity initially described in bacteria [56]. The overall immune memory of CRISPR/Cas9-based defense completes in three stages [9]. It commences with spacer acquisition by which the spacer (protospacer) sequence along with protospacer adjacent motif (PAM) is recognized and integrated into the CRISPR locus, followed by the expression stage during which CRISPR RNA (crRNA) and trans-acting crRNA (TracrRNA) are transcribed and finally the interference stage, in which the crRNA binds with the TracrRNA and forms a complex with Cas9 protein that is now ready for base-pairing and degradation of the target foreign DNA [57]. The components for genome-editing using CRISPR/Cas9 are a DNA endonuclease Cas9 protein and a customizable single-stranded guide RNA (sgRNA). sgRNA is a small non-coding RNA assembled by fusing crRNA and tracrRNA designed to edit a sequence adjacent to a PAM sequence [58]. The redesigning of crRNA (which is the case in single-stranded RNA-guided DNA nucleases) has been used to essentially targeting any DNA sequence in CRISPR/Cas9 system genome-editing in eukaryotes including crop plants [23]. Once the target DNA sequence is hybridized with the complementary sgRNA, high fidelity Cas9 triggers double-stranded DNA breaks (DSBs). The DSBs, introduced by CRISPR/Cas9 system, are repaired by cellular DNA repair pathways involving NHEJ, HR, or MMEJ, which ultimately result in the disruption of target genes due to the introduced indels [59]. As reviewed by Lee et al. [25], the latest developments with CRISPR/Cas9 has come so far with the possibility of multiplexing which enables the introduction of a package of multi-site mutations in the genome, dimerizing of the dCas9 (dead Cas 9) system fused to FokI nucleases for the sole purpose of silencing by binding (without cleavage), addition of a DNA-binding domain for improved specificity and splitting of Cas9 into two components for easy packaging and delivery.

The CRISPR/Cas adaptive immune system has gone through substantial improvements as variants of Cas proteins were discovered in recent years. A more simplified version of CRISPR/Cas-based genome-editing was reported after the characterization of type V Cas12a (formerly Cpf1) in *Francisella novicida* bacterium [60]. The three advantages of CRISPR/Cas12a over CRISPR/Cas9 genome-editing: staggered cutting, reliance on T-rich PAM, and requiring only crRNA (which does not require tracrRNA) made CRISPR/Cas12a system a more efficient, flexible, and simple sgRNA-DNA interference mechanism of genome-editing [61]. The latest characterization of type VI protein, RNA-guided RNase effector CRISPR/Cas13a (formerly C2c2) from the bacterium *Leptotrichia shahii*, has been designed to target ssRNA harboring protospacer sequence complementary to a single crRNA [62]. Overall, the application of CRISPR/Cas system for disease resistance development by either targeting the pathogen genome or host genes to interfere with susceptibility is more successful in the last couple of years due to simplicity in design, greater efficacy, high specificity, and almost universal applicability [11] (Table 1). The application of CRISPIR/cas9 is tremendous and more robust with high throughput manipulation of target genes. Some of the recent advancements in CRISPR/cas9-based genome-editing for the development of biotic and abiotic stresses include powdery mildew resistance in bread wheat [63], late blight resistance in potato [12], beet severe curly virus resistance [64], turnip mosaic virus resistance in *A. thaliana* [65], blast resistance in rice [66], cucumber vein yellowing virus [67], drought tolerance in maize [68], potassium deficiency tolerance in rice [69] (see review by Jaganathan et al. [70]).

**Table 1.** A summary of the applicability, complexity, and efficiency of genome editing tools used for disease resistance development in different plants.

Genome editing tool	Target sequence	Mutation to be introduced	Complexity	DNA repair mechanism	Plants exploited/experimental evidence	Efficiency
ZFN	Pathogenic viral genomes/replication protein binding elements	Frameshift	Most complex in applying for disease resistance development in plants	NHEJ/HR	*A.thaliana*[29,31] *N. benthamiana*[30]	Most efficient for smaller expression elements
TALEN	Effector/transcription factor binding elements	Nonspecifically, any mutation could be introduced	Complexity is reduced	NHEJ/HDR/HR	*O. sativa*[39–41] *N. benthaminana*[42]	Improved efficiency to be applied in plants
ODM	Sense/anti-sense-based plant genome sequence	Single base pair mutation	Decreased complexity with increased precision	Natural base pairing process	*A.thaliana*[71] *B. napus*[47] *Z. mays*[48] *N. tabacum*[43]	More efficient to be applied in plants
CRISPR/Cas	Guide ssRNA could be designed to target any target sequence	Mutation of various size can be introduced	Multiplexed and simplified	DSB DNA repair via NHEJ/ HR/MMEJ	*T. aestivum* [63] *A. thaliana*[65] *O. sativa*[66],[69] *C. sativus*[67] *Z. mays*[68]	Highest efficiency and universality for any target organism

## Achievements in molecular breeding for disease resistance by S gene editing in *Solanaceae*

Sustainable agricultural production to feed the projected population of 9.8 billion by 2050 posed an unprecedented challenge to plant breeders. Disease caused by bacterial and fungal pathogens contributes to 15% yield loss and the other 3% by viral pathogens [72], altogether exacerbating the demand for better breeding technologies for disease resistance. Of interesting phytopathogenic aspect is the cross-pathogenicity of most principal fungal and viral pathogens to potato, tomato, and pepper (Table 2), which urges the breeders for the development of interspecific, broad-spectrum, and durable resistance.

**Table 2.** Principal diseases of potato, tomato, and pepper.

Pathogen category	Causative agent	Target host	Disease conditioned (symptoms)	Reference
Bacterial	*Pectobacterium spp*. and *Dickeya spp.*	Potato, tomato and pepper	Blackleg and soft rot, black to brown discoloration of the stem	[73]
	*Pectobacterium carotovorum subsp. carotovorum (syn. Erwinia carotovora subsp. carotovora), Pectobacterium atrosepticum* and *Dickeya dianthicola (syn. Erwinia chrysanthemi)*	Mainly potato	Aerial stem rot, water-soaked lesion-like	[73]
	*Clavibacter michiganensis subsp. sepedonicus*	Potato and tomato	Ring rot	[73,74]
	*Streptomyces scabies, S. acidiscabies* and *S. turgidiscabies*	Potato and tomato	Common scab	[73]
	*Xanthomonas* *campestris*	Tomato and pepper	Bacterial leaf spot	[75,76]
Oomycete	*Phytophthora spp.*	Potato, tomato and pepper	Phytophthora root rot	[76,77]
Fungal	*Fusarium oxysporum*	Potato, tomato and pepper	Fusarium wilt	[77]
	*Verticillium spp.*	Potato, tomato and pepper	Verticillium wilt	[77]
	*Colletotrichum spp.*	Potato, tomato and pepper	Anthracnose	[76,77]
	*Alternaria solani*	Potato and tomato	Early blight	[77]
	*Septoria spp.*	Potato and tomato	Septoria leaf spot	[77]
	*Passalora fulva*	Tomato and pepper	Leaf mold	[77]
	*Oidium spp.*	Potato, tomato and pepper	Powdery mildews	[76,77]
	*Botryotinia fuckeliana*	Potato, tomato and pepper	Gray mold	[77]
	*Ralstonia* *solanacearum*	Potato, tomato and pepper	Bacterial wilt	[76,78]
Viral	*Alfalfa mosaic alfamovirus*	Potato, tomato and pepper	Necrosis and yellow mosaics	[77]
	*Capsicum mild mottle tobamovirus*	Pepper	Chlorosis and stunting	[77]
	*Cucumber mosaic cucumovirus*	Potato, tomato and pepper	Stunted growth and shoestring like appearance	[76,77]
	*Pepper mild mottle tobamovirus*	Pepper	Mottling, chlorosis, curling, dwarfing	[76,77]
	*Pepino mosaic potexvirus*	Tomato	Mosaic and chlorosis	[77]
	*Pepper veinal mottle virus (PVMV)*	Pepper	Mosaic, chlorosis, yellowing and stunting	[76]
	*Tomato spotted wilt tospovirus*	Potato, tomato and pepper	Leaf spots similar to early blight	[77,79]
	*Potato Y potyvirus*	Potato, tomato and pepper	Necrosis, mottling, mosaic and stunting	[77,80]
	*Tobacco mosaic tobamovirus*	Potato, tomato and pepper	Bright mosaic, interveinal yellowing, rigid leaves, mild mottling and stunting	[77,81]
	*Potato virus X*	Potato and tomato	Brown streaks on petioles or stems	[81,82]
	*Tomato chlorosis crinivirus*	Potato and tomato	Chlorotic mottling and interveinal yellowing	[77,83]
	*Tomato mosaic tobamovirus*	Tomato and pepper	Light and dark green mosaic in leaves	[77]
	*Tomato yellow leaf curl begomovirus*	Tomato	Stunting, leaf curling and yellowing	[77]
	*Pepper veinal mottle virus*	Pepper	Systemic interveinal chlorosis, mottle and distortion of abscission time and fruit	[76]

Most of the disease-resistant crop varieties (including the *Solanaceae*) are developed on the recognition-based dominantly inherited R genes; however, the novel recessive susceptibility mutant gene disease resistance developed by the genome-editing tools was found to be more durable [84,85] and associated with some fitness costs [11]. A list of diverse S genes silenced in the three *Solanaceae* crops either by genome-editing or RNA interference (RNAi) is summarized in Table 3. According to van Schie and Takken [86], S genes are grouped into three classes based on their contribution to susceptibility (Table 3). The first class is required for pathogen infection and penetration, including spore germination in spore-forming fungal pathogens. The conserved membrane-anchored protein-encoding orthologous genes such as mildew locus O (Mlo) in tomato, pepper, and other cereal crops are typical examples [87]. The second class includes negative regulators of plant immunity, also known as defense suppressors, which negatively regulate the expression of cellulose synthase genes such as CeSA3 [88]. The third class of S genes (such as SWEET genes) is involved in sugar biosynthesis and transport, which are required for pathogen sustenance and replication [89]. The conversion of the *Arabidopsis* eIF4E1susceptibility gene into resistance to *Clover Yellow Vein Virus (CYVV)* was possible by CRISPR/Cas9-cytidine base editor (CBE)-based genome-editing and even across plant species including the *Solanaceae* [90].

**Table 3.** List of selected disease-resistant *Solanaceae* crop plants developed by susceptibility gene-silencing.

S gene role[86]	S gene (contributing to susceptibility)	Protein product encoded	Plant species (host)	Disease conditioned	Pathogen	Off-target effect	Reference
Pathogen activation, penetration, sustenance and replication	*LeExP1*	Polygalacturonase and expansin (double mutant tested)	Tomato	Gray mold/rot	*Botrytis cinerea* (only fruit)	Reduced fruit softening	[91]
Pathogen activation and penetration, defense suppression	*Sitiens/Sit*	ABA aldehyde oxidase (Sitiens)	Tomato	Gray mold/rot, soft rot	*Botrytis cinerea, Erwinia chrysanthemi*	Increased sensitivity to drought, wilting (open stomata), impaired interaction of (beneficial) arbuscular mycorrhizal fungi, early germination	[92,93]
Pathogen activation and penetration	*SIMLO1 (Ol-2)*	Membrane anchored protein	Tomato	Powdery mildew	*Oidium neolycopersici, Leveillula taurica*	None reported	[94]
Pathogen activation and penetration	*CaMLO2*	Membrane anchored protein	Pepper	Powdery mildew, bacterial leaf spot	*Leveillula taurica, Xanthomonas campestris*	Reduced tolerance to drought stress	[94]
Pathogen activation and penetration, defense suppression	*Cel1*	Endo-beta-1,4-glucanase	Tomato	Gray mold/rot	*Botrytis cinerea* (only leaf phenotype, not fruit)	Increased sensitivity to biotroph (Pseudomonas), probable reduced fruit softening and reduced flower abscission.	[95]
Defense suppression	*CaWRKY1*	Transcription factor WRKY	Pepper	Pustule disease	*Xanthomonas axonopodis*	None reported	[96]
Defense suppression	*CaWRKY58*	Transcription factor WRKY (activator)	Pepper	Bacterial wilt	*Ralstonia solanacearum*	None reported	[97]
Pathogen sustenance and replication	*DMR1*	Homoserine kinase	Tomato	Powdery mildew	*Oidium neolycopersici*	Dwarfing	[98]
Defense suppression, decrease SA level	*SlDMR6-1 orthologue Solyc03g080190*	Downy mildew resistance 6	Tomato	Bacterial speck disease, root rot, bacterial spot	*Phythophthora Pseudomonas syringae, Xanthomonus spp.*	None reported	[113]
Pathogen sustenance and replication	*XSP10*	Lipid transfer protein	Tomato	Fusarium wilt	*Fusarium oxysporum f.sp. lycopersici*	None reported	[99]
Pathogen sustenance and replication	*UPA7*	Expansin	Pepper	Bacterial spot	*Xanthomonas campestris*	None reported	[100]
Pathogen sustenance and replication	*UPA20*	bHLH Transcription factor, induces expression of UPA7	Pepper (*C. annuum*)	Bacterial spot	*Xanthomonas campestris*	None reported	[100]
Pathogen sustenance and replication	*eIF4E1*	Eukaryotic (translation) initiation factor *eIF4E*	Tomato (*S. lycopersicum*)	Potyviruses	*PVY, TEV, PepMoV, ERV, PepSMV, PepYMV, PVV (Potato virus Y, Tobacco etch virus, Pepper mottle virus, Equadorian rocotto virus, Pepper severe mosaic virus, Pepper yellow mosaic virus, Potato virus V)*	Plants are smaller (RNAi targets both copies), not effective against 4 non potyvirus strains	[101]
Pathogen sustenance and replication	*pvr1*	Eukaryotic (translation) initiation factor *eIF4E*	Pepper (*C. chinense*)	Potyviruses	*PepMoV, PVY, TEV (Pepper mottle virus, Potato virus Y, Tobacco etch virus)*	None reported	[102]
Pathogen sustenance and replication	*pvr2*	Eukaryotic (translation) initiation factor *eIF4E*	Pepper (*C. annuum*)	Potyviruses	*TEV, PepVMV, ChiVMV, PVY (Tobacco etch virus, pepper veinal mottle virus, Chili veinal mottle virus, Potato virus Y)*	None reported	[103]
Pathogen sustenance and replication	*pvr6*	Eukaryotic (translation) initiation factor *eIF4E* and *eIF*(iso)*4E*	Pepper (*C. annuum*)	Potyviruses	*PVMV, ChiVMV (Pepper veinal mottle virus, Chili veinal mottle virus)*	None reported	[118]
Defense suppression	*CESA3*	Cellulose synthase	Potato	*Phytophthora infestans*	Late blight	None reported	[108]
Pathogen sustenance and replication	*DMR6*	Salicylic acid 5-hydroxylase	Potato	*Pseudomonas syringae*	*Bacterial brown spot/bacterial speck*	None reported	[108]
Pathogen sustenance and replication	*DMR6*	2-oxoglutarate (2OG)-Fe (II) oxygenase	Potato	*Phytophthora infestans*	Late blight	None reported	[12,13]
Pathogen sustenance and replication	*DND1*	RNA-binding protein	Potato and tomato	*Pseudomonas syringae*	*Bacterial brown spot/bacterial speck*	Dwarfing, autonecrosis, color loss	[104,108]
Defense suppression	*SR1*	Truncate SR1 protein, calmodulin-binding transcription activator	Potato	*Podophaera fusca*	*Powdery mildew*	None reported	[108]
Pathogen activation and penetration	*PMR4*	Cellulose synthase	Potato	*Podophaera fusca*	*Powdery mildew*	None reported	[108]
Bacterial activation and penetration	*BIK1*	Ser/thr protein kinase	Potato	*Pseudomonas syringae*	*Bacterial brown spot/bacterial speck*	None reported	[108]
Defense suppression	*CPR5*	Unknown	Potato	*Pseudomonas syringae, Peronospora parasitica*	*Bacterial brown spot/bacterial speck, downy mildew*	Dwarfing, color loss	[108]
Defense suppression	*DND2*	Dead-end protein	Potato	*Phytophthora infestans*	*Late blight*	None reported	[108]
Pathogen sustenance and replication	*PMR5*	Pectate esterase (probably)	Potato	*Erysiphe cichoracearum*	*Powdery mildew*	None reported	[108]
Pathogen sustenance and replication	*PMR6*	Pectate lyase	Potato	*Erysiphe cichoracearum*	*Powdery mildew*	None reported	[108]

Potato, as one of the staple foods worldwide, has been under genome-editing with the objective of disease resistance, nutritional improvement, and reduced herbicide susceptibility [105–107]. Using *A. thaliana* reference genome, many orthologous S genes were identified in potato paving a way for genome-editing for the development of disease resistance that could be reproduced across crop species (Table 3) [108]. It was demonstrated that RNAi-based silencing of six different S genes conferred resistance against potato late blight disease by knocking down the expression of multiple S genes [13]. Moreover, such RNAi-based impairments of orthologous S genes could be extrapolated to any of the genome-editing tools for the development of multiple disease resistances with low or no pleiotropic effects as they are mainly plant-species-dependent [108]. As some pathogens target host immunity through ubiquitination, ubiquitin ligase gene knockout has led to an increased resistance against *Phytophthora infestans* in potato [109]. The application of genome-editing for the development of disease resistance in crops is a two-way approach as the same mechanism of editing S genes of the host could also be applied to editing the genome of the pathogenic RNA viruses with CRISPR/Cas13a effector nucleases targeting viral RNA. Disease symptoms and accumulation of Potato Virus Y (PVY) were successfully suppressed in transgenic potato lines transformed with Cas13a/sgRNA with high efficiency which could be customized to interfere with multiple strains of PVY [110].

One of the most robust and durable disease resistance developments in tomato by deterring pathogen penetration was conferred by the mutation in mildew locus O (Mlo), an S gene that encodes a membrane-associated protein conserved in both monocots and dicots [86,111]. A more fascinating breakthrough was achieved by the development of transgenic-free powdery mildew-resistant tomato variety in less than a year by editing SlMlo1 using the CRISPR/Cas9 system [112]. A CRISPR/Cas9 system-based genome-editing has demonstrated the successful introduction of an induced mutation into SlDMR6-1 gene, that is up-regulated during the infection by different pathogens. A small deletion mutation in the gene resulted in a truncated protein due to frameshift mutation, which triggered elevated salicylic acid levels leading to disease resistance against *P. syringae, P. capsici*, and *Xanthomonus* spp. [113]. A broad-spectrum resistance to powdery mildew (caused by *Oidium neolycopersici*) conferred by Ol-2 gene has also been developed by the loss of Mlo function using viral vector delivery [114], which could potentially be more exploited by the CRISPR/Cas9 system. Likewise, CRISPR/Cas9 was used to develop bacterial speck disease-resistant tomato with no detected defense trade-off by editing the SlJAZ2 gene [115]. As viruses are attributed to significant yield loss to vegetables, including tomato, mitigation of viral infections and subsequent symptom development has been another area of viral genome-editing. A CRISPR/Cas9 system-mediated viral genome-editing by disrupting the intergenic sites has resulted in significantly reduced accumulation of tomato leaf yellow curly virus DNA and other DNA viruses [116]. A site-directed mutation introduced to 4E (eIF4E) gene by CRISPR/Cas9-based system has demonstrated enhanced and heritable resistance to pepper mottle virus (PepMoV) in tomato [117].

The cap-binding protein (also known as eukaryotic translation initiation factor 4E (eIF4E)) encoding gene is one of the components of susceptibility as it plays an essential role in the infection cycle of potyviruses in peppers and other crops. Disrupting the eIF4E encoding genes with CRISPR/Cas9 has successfully broken its interaction with 5-terminal protein (viral protein genome linked protein) and triggered potyvirus resistance in chili pepper and many other crops [11,118]. A C-T base conversion editing tool (CBE) associated with CRISPR/Cas9 was applied to edit a transcription factor NAC72 encoding gene resulting in the anthracnose resistance in chili pepper [119]. CRISPR/Cas9-mediated sequence-specific mutation of eIF4E1 gene has also led to the development of PepMoV resistant transgenic-free tomato [120], reiterating the potential of this method as a gateway to create a mutation on a single gene for the development of multiple virus resistances by deploying the multiplexed CRISPR/Cas9 system. A mutant escape in a single site targeted CRISPR/Cas9 was overcome by constructing duplex and triplex CRISPR/Cas9 constructs that target the viral genome at two or more sites simultaneously and has shown the potential of this approach to eliminate mutant escape and total elimination of chili leaf curl virus (ChilLCV) DNA in *Nicotiana benthamiana* [121].

The molecular characterization and mechanism of action in conditioning susceptibility conferred by S genes are less understood than the R-gene counterparts. Molecular identification and characterization of S genes have been an emerging area of research as the development of durable and broad-spectrum disease resistance has been demonstrated to be more feasible with genome-editing tools, especially CRISPR/Cas-mediated genome-editing. We mined 26 susceptibility-related genes sequenced and characterized in potato, tomato, pepper, and their orthologs in *Arabidopsis* (Table 3). Among the listed S genes, the majority (65.38%) were found with no off-target effects, which is often the main collateral constraint in S genome-editing for disease resistance breeding. To have a broader picture of the biological role of S genes in inducing susceptibility, the sequences were re-annotated (Figure 1; Supplemental material). The molecular function of the majority (61.5%) of the S-related genes was either metal ion-binding, transcription, or translation factors to vigorously modulate pathogenicity and eventually obstruct the host defense system (Figure 1). Interestingly, there are some S genes involved in defense response and systemic acquired resistance to bacterial and fungal pathogens. In *Arabidopsis,* it was reported that mutation in the nucleotide-binding leucine-rich repeat (NB-LRR) R gene families has led to the development of susceptibility to fungal victoria blight disease [10]. Nearly one-third (30.76%) of the characterized S genes in these crops are membrane components (Figure 1 C) or in a more broad category, 76.92% are attributing to cellular anatomy (Figure 1 D). It indicates that these membrane-anchored S gene products are likely involved in the process of pathogen infection and pre-penetration processes such as spore germination. In maize, for instance, conidial germination and appressorial differentiation of powdery mildew conditioning fungus *Blumeria graminis* was impaired in wax mutant *glossy11* regenerated plants [122]. One of the astonishing reports in disease resistance was the loss-of-function mutation in the membrane-bounded S gene, Mlo, first identified in barley [123]. Mlo-mediated resistance, which conferred a broad-spectrum version of powdery mildew resistance, was also induced in tomato and other crops [114].
**Figure 1.** Susceptibility gene annotation and GO count. mined S genes were re-annotated and directly counted for BP (a), MF (b), CC (c) and summary of top GO distribution (d) in the three categories as analyzed by BLAST2GO [73]; BP, biological process; MF, molecular function; CC, cellular component; GO, gene ontology. E-value cutoff of 1e-05 or less was considered for annotation while default setting was used for the all the other parameters.

**Figure 1.** (Continued)

## Conclusion

Disease resistance is typically conferred by dominantly inherited genes characterized by their recognition by single-pathogen-derived molecules, which could eventually likely to be overcome and turn the host susceptible over time. A more durable and broad-spectrum disease resistance tool has recently emerged by either targeting the transcripts or the genes of susceptibility proteins of the host or the genes of the pathogens. As the S genes are functionally conserved across plant species, S-related genes and/or their orthologous genes-editing in economically important vegetable crop plants such as potato, tomato, and pepper could have a paramount significance in developing durable and broad-spectrum disease resistance. As many off-target effects are reported in S-gene silenced lines, it has to be well established before commercialization of such crops. Moreover, as far as the cellular localization of S-genes are concerned, many of the S-genes are cell membrane associated which are involved in the process of infection prepenetration and/or spore germination. The latest genome-editing tools such as multiplexed CRISPR/Cas with enhanced precision for site-specific genome-editing have led to the substantially improved speed of breeding cycles. Moreover, the variants of genome-editing tools have brought many insights into the molecular mechanisms of susceptibility and site-specific mutagenesis. Genome-editing-based transgenic-free disease resistance development has also eased the hurdles surrounding the regulations and ethical issues of genetic engineering.

## Supplementary Material

Supplemental Material

## Data Availability

All the data that support the analysis of the present paper can be available upon reasonable request from the corresponding author.

## Future prospects

Genome-editing has presented unprecedented precision and high throughput manipulation of complex genomes which are the main tackles in classical and molecular breeding. Since the first generation of genome-editing with ZFN, CRISPR/Cas variants are now enabling editing of virtually any sequence of interest for different breeding objectives as the genomes of almost all crop plants are sequenced and openly accessible. Despite all the endeavors so far, however, the off-target effects are the main hurdle characterizing S gene editing for the development of disease resistance. The next decade is expected to see a high throughput identification of pleiotropic genes and alternative genome-editing approaches such as targeting S genes with minor off-target effects. The use of tissue or temporal specific promoters in multiplexed CRISPR/Cas gene construct could also minimize the off-target effects associated with yield and other important agronomic traits.
